The article "An Initial Study on Automated Acupoint Positioning for Laser Acupuncture" was published in 2022. Journal: Evid Based Complement Alternat Med.

# An Initial Study on Automated Acupoint Positioning for Laser Acupuncture

**DOI:** 10.1155/2022/8997051

**Published:** 2022-08-22

**Authors:** Kun-Chan Lan, Chang-Yin Lee, Guan-Sheng Lee, Tzu-Hao Tsai, Yu-Chen Lee, Chih-Yu Wang

**Affiliations:** ^1^Department of CSIE, National Cheng Kung University, Tainan 701, Taiwan; ^2^The School of Chinese Medicine for Post-Baccalaureate, I-Shou University, Kaohsiung 824, Taiwan; ^3^Department of Chinese Medicine, E-DA Hospital, Kaohsiung 824, Taiwan; ^4^Graduate Institute of Acupuncture Science, China Medical University, Taichung 404, Taiwan; ^5^Department of Acupuncture, China Medical University Hospital, Taichung 404, Taiwan; ^6^Department of Biomedical Engineering, I-Shou University, Kaohsiung 824, Taiwan

## Abstract

Acupuncture plays an important role in traditional Chinese medicine (TCM) and is one kind of an inexpensive and effective treatment. However, some people might be reluctant to receive acupuncture treatment due to fear of pain. Laser acupuncture, thanks to its painless and infection-free advantages, has recently become an alternative choice to traditional acupuncture. The accuracy of acupuncture point positioning has a decisive influence on the quality of laser acupuncture. In this study, built on top of our prior work, we proposed a low-cost automated acupoint positioning system for laser acupuncture. By integrating several machine learning algorithms and computer vision techniques, we design and implement a robot-assisted laser acupuncture system on top of a smartphone. Our contributions include the following: (a) development of an effective acupoint estimation algorithm with a localization error less than 5 mm; (b) implementation of a smartphone-controlled automated laser acupuncture system with lift-thrust function, as a point-of-care device, that can be used by patients to relieve their symptoms at home.

## 1. Introduction

Traditional Chinese medicine (TCM) is one kind of medicine based on more than 2000 years' clinical practice covering both diagnosis and treatment of diseases. In TCM, acupuncture plays a very important role and has unique advantages and significant clinical values. Its efficacy has been confirmed by many studies [1, 2]. Recently, thanks to its painless and noninvasive nature, laser acupuncture has become an alternative to traditional acupuncture and many studies have shown its effectiveness [3–6].

In our previous work, a novel laser acupuncture instruments with the lift-thrust function have been developed [7, 8]. Specifically, the lift-thrust function of laser acupuncture is implemented by moving the focused laser spot back and forth. The energy of the laser is concentrated at the focused light spot, which is considered as the tip of an acupuncture needle. When the laser light enters the human body, the position of the focused light spot is mobile, as if the needle tip is moving through the acupuncture point, thereby realizing the lift-thrust function of the laser acupuncture.

We demonstrated that the laser acupuncture with the lift-thrust function performs better than the traditional laser acupuncture in our prior work [9]. In particular, the laser power used in our system is relatively lower compared with that in most of the commercially available laser acupuncture instruments. Lower power allows for a longer stimulating time, which is consistent with the practice of “needle retention” in traditional acupuncture. On the other hand, a longer stimulating time suggests that acupuncture practitioners have to hold the laser acupuncture instrument (which is much heavier than a steel needle) for a longer time, which might not be convenient for clinical practice. Considering the physical labor paid by the acupuncturist, it is natural to restore to a robot to improve the efficacy of therapy. Motivated by this need, we propose a robot-assisted laser acupuncture system which consists of three parts: a smartphone-based chatbot, an acupuncture point database, and an acupoint positioning system. The chatbot app is implemented based on the popular BERT model [10]. For the acupoint database, we reuse a database we built in our previous study [11]. In this paper we focus on describing automated acupoints positioning which is the core of our proposed system.

To the best of our knowledge, this is the first prototype system that has been developed for smartphone-controlled automated laser acupuncture. The remainder of this paper is organized as follows: Section 2 discusses the related work. We describe our methods in Section 3.  Section 4 discusses our experiments and results. Some observations are presented in Section 5. Finally, we conclude this paper in Section 6.

## 2. Related Work

Traditionally, TCM doctors rely on some methods such as bone measurements, body surface marker, and cun measurements to locate various acupoints [12]. However, it is difficult to remember the locations and corresponding therapeutic effects of all the acupoints (more than 400) without extensive training. On the other hand, acupoints are generally situated along meridians which are high-conductivity channels on the skin [13]. The Ryodoten, or electropermeable points (EPP), are a series of points with higher electrical conductivity than other areas of the skin [14]. These points are found to be close to the acupoints on meridians recognized in Chinese medicine. Inspired by this observation, many acupoint localization instruments were built based on the electrical characteristics of acupoints (i.e., looking for areas with a lower skin impedance to estimate the location of acupoints). However, such a contact-based acupoint searching method has some disadvantages such as a longer search time, inconvenient operation, and the inability to locate all the acupoints at the same time. In contrast to the method, based on skin conductivity, an image-based acupoint positioning method has the advantages of real-time localization, user-friendliness, and simultaneous positioning.

As far as we know, the image-based acupoint positioning system is currently still an underexplored area of research. Lin [15] used the landmark points on the back contour to localize the spine points based on the concept of barycentric coordinates. Given that the locations of acupoints on the back are relative to the positions of spine points, back acupoints can be localized once the positions of spine points are correctly identified. Jiang et al. proposed acu glass [12] for acupoint localization and visualization. They created a reference acupoint model for the frontal face, and the acupoint coordinates are expressed as a ratio to the face bounding box (computed by the face detector). The reference acupoints are rendered on top of the input face based on the height and the width of the subject's face and the distance between the eyes, relative to the reference model. They used ORB feature descriptors to match feature points from the current frame and the reference frame, to get the estimated transformation matrix. Instead of scaling the reference acupoints such as the study in [12], Chang and Zhu [16] implemented a localization system based on cun measurement. Cun is a traditional Chinese unit of length (its traditional measure is the width of a person's thumb at the knuckle, whereas the width of two forefingers denotes 1.5 cun and the width of four fingers side-by-side is three cuns). They used the relative distance between landmarks to convert pixel into cun. The acupoint can be located based on its relative distance (in cun) from some landmark point. There are some issues with the abovementioned approaches for acupoint localization, such as that the differences of the body shape between different people are not considered. Recently, Chen et al. designed and implemented a system to localize facial acupoints on a smartphone by utilizing the 3D morphable model (3DMM) and achieved a localization error of 2.4 mm [17]. In this work, we adopt a similar approach as [17] for the acupoint point positioning in the image space.

Acupuncture is gaining increasing interests with the emergence of integrative medicine. Traditionally, acupuncture is performed by a licensed acupuncturist. It is natural to resort to a robot for such a labor-intensive job for its precision and endurance. In a robot-assisted acupuncture system, the camera and the robot arm are the main components. In such a system, one first determines the positions of acupoints in the image space, and then moves the robot arm to the position where the camera sees to perform the acupuncture. Therefore, it is important to know the relationship between the image space and the robot arm space. In literature, the problem of determining this relationship is referred to as the hand-eye calibration problem which is to solve a matrix equation of the form *Y* = *XM* [18]. In our case, *Y* is the coordinate of the robot end-effector (in the robot arm space), *X* is the coordinate of an acupoint (in the image space), and *M* is the unknown transformation between the robot arm space and the image space. In robotics, this is a well-known problem and many approaches have been proposed [19, 20]. In practice, there are two different ways for hand-eye calibration depending on where the camera is placed: hand-in-eye and hand-to-eye calibrations. Hand-in-eye refers to the calibration where the camera is mounted on the robot arm and therefore the camera will move as the robot arm moves. Potentially, the viewing space of the camera will be limited by the operating range of the robot arm. On the other hand, hand-to-eye refers to the calibration where the camera is statically placed at a position independent of the movements of the robot arm. This generally will provide a macroscopic way of the environment. In this work, we design our system with the hand-to-eye method since that allows a viewing space of the camera which can cover the whole acupuncture area. In addition, we adopt the perspective transformation [21] to solve the hand-eye calibration problem.

Lifting and thrusting is an important manipulation method in traditional acupuncture. After piercing the skin to a certain depth, practitioners repeatedly move the tip of the needle vertically at a specific frequency to stimulate the skin, fascia, fat, muscles, and other tissues [22]. With lift and thrust operation, specific effects such as reinforcement and reduction might be achieved during the acupuncture process. In our previous work, laser acupuncture instruments with the lift-thrust function have been developed [7, 8]. Furthermore, we also showed that laser acupuncture with lift-thrust operation enabled a more rapid, stable, and lasting temperature rise of the fingertip than that without the lift-thrust operation [9]. In those studies, the lift-thrust function of laser acupuncture is implemented by moving a focused laser spot back and forth with an electrical micro-activator and mobile lens. In the current study, we would like to emulate the lift and thrust operation by the moving robot arm (up and down) with a fixed focal length laser.

## 3. Methods

Our automated acupoint positioning system includes two parts: (A) image-based acupoints localization; (B) hand-eye calibration which consist of two processes: transformation matrix calculation and coordinate transformation. The purpose of transformation matrix calculation is to find the relationship between the camera space and the robot arm space. This process only needs to be performed once when initially setting up the system. As shown in Figure 1, the camera first reads an image as the input and passes it to the acupoint estimation process to get coordinates of the acupuncture points in the image space. Second, the obtained image coordinate is passed to the coordinate transformation process to get coordinates of the acupoints in the robot arm space. Finally, the computed robot arm coordinate of the acupoint is used to position the robot arm to perform automated laser acupuncture.

### 3.1. Image-Based Acupoint Localization

In our previous work, we have established an image-based acupoint localization method for locating face acupoints with a smartphone camera [23]. In this work, we adopt a similar approach with some modification, as shown in Figure2 (localization of hand acupoints is used here as an illustration for explaining our method). Specifically, to improve the speed and accuracy of the image recognition process, we replace the homography transformation (HOG) method [21] used in our prior work [23] with the convolutional neural network (CNN) technique [24], based on MobileNet [25], to detect the region of interest (ROI) area (i.e., the area that contains the acupoints). Furthermore, we implemented the constrained local Method (CLM) [26] for the landmark detection. The CLM methods, estimating landmark locations *x* based on the global shape patterns of objects as well as the independent local appearance information around each landmark, are comparatively faster than the regression tree method [27] used for landmark detection in our prior work [23]. As shown in Figure 3, our acupoint estimation procedure consist of two parts: an offline process and an online process, which are discussed next.

#### 3.1.1. Offline Process

In the offline process, we first manually collect the 2D hand image data from different sides (front and back) of the hand using the smartphone camera. These data will be used to train a MobileNet model as well as create a hand landmark model for the hand detection and landmark detection tasks in the online process later. In addition, we employ the 3D scanner to create a 3D hand model and annotate the landmark points and acupoints on this model to facilitate the pose estimation and acupoint estimation tasks in the online process. Conceptually, the aim of this offline process is to use the collected 2D/3D image data (from a number of subjects) to create a “virtual” acupuncture dummy model (in this case, for the hand) as a reference model, on which the acupoints are annotated. Therefore, in the online process we can match the input image (from the user) with this reference model to estimate the acupoints in the input image. This idea of matching the input image to the reference model is theoretically similar to the learning process of how a person finds the locations of acupoints on his/her body through an acupuncture dummy.

#### 3.1.2. Online Process

The hardware components of our system consist of a smartphone and a robot arm. The smartphone is mounted above the robot arm as shown in Figure 1. The smartphone is used to localize the acupoint and direct the movement of the robot arm to the desired location for the laser stimulation.

In the online process, the hand in the input image is first detected by the pretrained MobileNet model from the offline process. The hand detection process will output a region in which the hand is located. The landmarks on the hand are then identified through a CLM method [26] based on ORB [28] and RANSAC [29]. The hand pose can then be estimated by matching the detected landmarks on the 2D input image and the annotated landmarks on the 3D model. Once the hand pose is determined, the 3D model can be aligned with the 2D input image and projected to the 2D space. Finally, the acupoint estimation problem can be treated as an image deformation process [23]. In the process the detected landmarks (in the 2D input image) and the annotated landmarks (on the 3D model, and now projected to the 2D space) are used as the control points to estimate the acupoints in the input image by deforming the annotated acupoints on the 3D model (which are now projected to the 2D).

### 3.2. Hand-Eye Calibration

Once the coordinates of the acupoints are estimated, the next step is to move the robot arm (carrying the laser acupuncture device) to the located acupoint position. This involves converting a 2D coordinate in the image space to its corresponding 3D position in the robot-arm space, the so-called hand-eye calibration. In this work, we first move the robot arm to the position that corresponds to the calculated image coordinate on the *x*-*y* plane. Then, we move down (along the *z*-axis) the robot arm to reach the acupoint using a height sensor. Therefore, the transformation from an image coordinate to a robot-arm coordinate can be performed in 2D. Here the perspective transformation [21] is used in our system to transform coordinates between two 2D planes, which can be expressed by the following formulas:

(1) $$\begin{array}{c} X=\frac{ax+by+c}{gx+hy+1},\\ Y=\frac{\text{d}x+\text{e}y+f}{gx+hy+1}. \end{array}$$

In the equation, (*x*, *y*) is the source coordinate (the image coordinate in our case) and (*X*, *Y*) is the target coordinate (i.e., the robot-arm coordinate). The eight parameters (*a*∼*h*) can be estimated to control in-plane-rotation, out-plane-rotation, scaling, shearing, and translation between source and target coordinates. To balance the computation time and accuracy.

In this work we randomly selected 13 reference points (which were taken at a specific height) to solve the perspective transformation equation based on the least square method [30]. Here, we can model these estimated parameters (i.e., *a*∼*h*) as a perspective matrix *T* so that (*X*, *Y*) = *T∗*(*x*, *y*).

Note that given that the reference points were selected from the *x*-*y* plane at a specific height (which is referred to as the “calibration height”) and the target acupoint could locate at a different height (i.e., higher or lower than the calibration height, as illustrated in Figure 3), errors will occur if we do not consider this height difference. We resolve this issue by performing another perspective transformation to convert the image coordinate obtained at height *b* to the image coordinate at height *a*, as shown in the equation (2), which is referred to as the “height fine-tuning process” in this paper. Here *P*_*a*_^″^  is the image coordinate at height *a*, *P*_*b*_^″^ is the image coordinate at height *b*, and *F* is the perspective matrix. To compute *F*, we collect another set of reference points from the *x*-*y* plane 1 cm higher than the calibration height to solve the linear equations. Finally, by combining the two perspective transformations described previously, we can now obtain an equation as shown in equation (3) to transform the estimated image coordinate of the acupoint to a robot-arm coordinate for positioning the laser acupuncture. Here *p*_*i*_^″^ is the estimated image coordinate of the acupoint, *p*_*i*_′ is the robot-arm coordinate, and *k* is the height difference between the acupoint and the calibration height, which can be estimated by the height sensor.

### 3.3. Evaluation of the Proposed System

Several sources of errors could affect the performance of our proposed system in positioning the laser acupuncture. The contributing factors to the robot-arm positioning accuracy include the accuracy of estimating the acupoint coordinate (in the image space), the transformation from the image coordinate to the robot-arm coordinate, the height fine-tuning process, and the possible mechanical error of the robot arm.

#### 3.3.1. Evaluation of the Accuracy of Acupoint Localization in the Image Space

In our experiment, 18 acupoint on the right hand were selected for evaluating the accuracy of acupoint estimation. The acupoints are listed as follows:

  Back of the hand: LU-11, LI-1, LI-2, LI-3, LI-4, SJ-1, SJ-2, SJ-3, SI-1, SI-2, SI-3, SI-4, and HT-9
  Palm: LU-10, PC-8, PC-9, HT-8, and HT-7

Ten young adults with ages ranging from 20 to 30 years are recruited and their data is used to train the AI models, as shown in Figure 3. The 18 selected acupoints are first marked with 5 mm diameter stickers served as the ground truth. Given that there is no consensus about the shape and the size of acupoint in the literature [31] (for example, a study examined the size of 23 acupoints and reported significant variability from 2.7 to 41.4 cm [32]), here, we follow the suggestion of some prior work [33–35] and conservatively choose the size of 5 mm which is smaller than most of the reported sizes from the literature. The smartphone is placed above the hand 30 cm from the hand. The estimation error is defined as the distance between the estimated position and the center of the sticker. This experiment was approved by the Institutional Review Board (IRB) of E-DA Hospital, Kaohsiung, Taiwan (IRB number. EMRP-105-005 (RIV)).

#### 3.3.2. Evaluation of the Accuracy of Hand-Eye Calibration

To evaluate the errors introduced by the transformation from the image coordinate to the robot-arm coordinate, we placed a plate on a desk, randomly selected 9 points on this plate, and marked their positions with stickers. We then identified the image coordinates of these selected points, and they are as follows: (240,160), (320,160), (400,160), (240,240), (320,240), (400,240), (240,320), (320,320), and (400,320). Next, the image coordinate of the selected point was transformed into the robot arm coordinate using equation (1). The robot arm then moved to the computed coordinate. Finally, we calculate the distance between the tip of the robot arm and the sticker, and this distance is defined as the hand-eye calibration error.

#### 3.3.3. Evaluation of the Accuracy of the Height-Fine-Tuning Process

To evaluate the accuracy of the height-fine-tuning process, the same test points discussed previously are used. Again, we first identified the image coordinates of the test points at different heights (from the plate) in advance as the ground truth. We then moved the robot arm to the computed coordinate based on equation (2). Finally, we compute the distance (in the image space) between the tip of the robot arm and the ground truth, and this is defined as the height-fine-tuning error.

#### 3.3.4. Evaluation of the Accuracy of Localization of the Proposed Robot-Assisted System

The localization accuracy of the proposed robot-assisted system depends on the performance of the abovementioned three processes. For its evaluation, we further recruited five subjects (who are not included in our training data) to evaluate the accuracy of the proposed system.

#### 3.3.5. Effect of Laser Acupuncture with Lift-and-Thrust Operation on Pulse Amplitude and Pulse Rate Variability (PRV)

Based on the proposed robot positioning system, we now can emulate the lift-and-thrust operation [9] by moving the robot arm (up and down) with a fixed focal length laser. We compared the effects of traditional steel needle acupuncture (performed manually) and laser acupuncture (with the aid of our proposed system) on the response of the human body. Three different acupuncture stimulation methods were compared: (a) laser acupuncture without lifting-thrusting function; (b) laser acupuncture with lifting-thrusting function; (c) traditional acupuncture stimulation (without lifting-thrusting operation).

The experiments were proceeded as follows: 10 healthy subjects (five males and five females) were recruited. Each subject received the abovementioned three types of stimulation for 5 minutes at Neiguan and Hegu points on both hands separately (at least 24 hours apart for each experiment). Photoplethysmography (PPG) signals (from the subject's wrist) were measured before and after the stimulation (the unit of PPG waveform is measured in mV). The PPG data were used to estimate the changes in pulse amplitude and pulse rate variability (PRV). Prior studies have found the changes of pulse amplitude and PRV can be associated with various diseases [36–40]. For example, changes in pulse amplitude and PRV have been found in patients with sleep apnea [36, 40]. The sampling rate of the PPG data is 25 Hz and the duration of the measurements is five minutes. To detect the pulse wave systolic peak (PWSP), we implemented an algorithm based on an event-related moving average [41]. Once the pulse wave peaks are identified, peak-to-peak (PP) intervals can then be computed and the power spectrum of the PP tachogram can be obtained. In this work, the PRV is computed as the power in the high frequency range (i.e., HF). The purpose of detecting the HF power is to observe the activity of the parasympathetic nerve, so as to know whether the autonomic nerve will be in a relatively relaxed state after laser acupuncture stimulation.

(2) $$\begin{array}{c} P_{a}^{\prime \prime }=F*P_{b}^{\prime \prime }, \end{array}$$

(3) $$\begin{array}{c} p_{i}^{\prime }=Tp_{i}^{\prime \prime }\left(KF-K+1\right). \end{array}$$

## 4. Results and Discussion

In this section, we present the results for the evaluation of sources of errors that could affect the performance of our proposed system, including the accuracy of estimating acupoint coordinate (in the image space), the transformation from the image coordinate to the robot-arm coordinate, and the height fine-tuning process.

### 4.1. The Accuracy of Acupoint Estimation in the Image Space

As shown in Figure 4, the average error is about 2 mm. The variations in the estimation errors might be due to the fact that while the subjects were asked to open their fingers during the acupoint estimation process as shown in Figure 3, different subjects might open their hands with various degrees, which results in the variations in the landmark detection errors.

### 4.2. The Accuracy of Hand-Eye Calibration

Figure 5 shows the errors for various test points, and the average error is about 0.5∼0.6 mm. The variations in errors for various test points might be due to the fact that our selected reference points are not evenly distributed in the image space.

### 4.3. The Accuracy of the Height-Fine-Tuning Process

As shown in Figure 6, the height-fine-tuning error is about 0.1∼0.2 mm on average, which is comparatively much smaller than the errors introduced by the acupoint localization and coordinate transformation processes.

### 4.4. The Accuracy of Acupoint Positioning of the Proposed System

The average positioning error of our proposed system is about 3.4 mm, as shown in Figure 7(a). In addition, we find that the acupoint estimation process accounts for most of the positioning error (>60%) for most acupoints, as shown in Figure 7(b). In addition, we observe that some of the selected acupoints (such as LU-11) appear to have a larger acupoint estimation error as compared to the results from the training data (as shown in Figure 4), which suggests a sign of overfitting (probably due to the small sample size of our training data). We plan to improve this in our future work.

### 4.5. Effect of Laser Acupuncture with Lift-and-Thrust Operation

Figure 8 shows the changes in pulse amplitude and PRV before and after needle and laser stimulation. Some observations are found as follows: (1) as compared to laser acupuncture, larger changes in both pulse amplitude and PRV have been observed for the needle acupuncture, for both Hegu and Neiguan acupoints.

(2) Laser acupuncture with lifting-thrusting function produced a larger increase in both pulse amplitude and PRV than that without the lifting-thrusting function. Note that in most cases, our proposed automated laser acupuncture system (with lifting-thrusting operation) has a performance (demonstrated by the increase of pulse amplitude and PRV) close to that of needle acupunctures which were performed manually.

There are several limitations in this work. First, the sample size of test subjects is small in this study, which might not be able to cover the heterogeneity among people (e.g., skin color, body shape, etc.). Second, due to the limitation of time and space, in this paper, we only evaluate the positioning accuracy of hand acupoints. Third, given the increasing popularity of depth-camera-equipped smartphones, the height-tuning process could be removed from our positioning system when a depth-camera-enabled smartphone is employed. In addition, we currently detect the depth of the hand using a height sensor mounted on the robot arm. Such a sensor might not be necessarily needed when a depth camera is available. These limitations will be improved in our future work. In addition, we plan to conduct clinical research with the proposed system in the future and demonstrate the results of our research through medical statistical methods.

## 5. Conclusion

In this work, we proposed a smartphone-based automated acupoint positioning system for laser acupuncture with lifting-thrusting operation, based on the integration of several machine learning methods and computer vision techniques. There are three main contributions in the present research. First, we successfully implemented a mobile phone-controlled automatic laser acupuncture device based on a robotic arm. Second, the established system achieved an accuracy with a <5 mm of average acupoint positioning error. Third, it is verified that the automatic laser acupuncture combined with the lifting and thrusting function can significantly improve its efficacy in affecting the pulse amplitude and pulse rate variability compared with that without the lifting and thrusting function.

## Figures and Tables

**Figure 1:** The architecture of the proposed system.

**Figure 2:** Flow chart of acupoints estimation.

**Figure 3:** Errors caused by different heights.

**Figure 4:** Estimation errors for various acupoints.

**Figure 5:** Hand-eye calibration errors for various test points.

**Figure 6:** Height-fine-tuning error for various test points.

**Figure 7:** The positioning errors for each acupoint and the contribution by different sources of errors. (a) The positioning error for each acupoints. (b) The contribution by various sources of errors.

**Figure 8:** Changes in pulse amplitude and pulse rate variability (PRV), the unit (*y*-axis) of PRV is in 100 ms^2^.

## Data Availability

No data were used to support this study.
